# Correlation Analysis of CML, sRAGE, and esRAGE and the Measure of Atherosclerosis of Coronary Heart Disease

This article has been retracted.

**DOI:** 10.1155/2022/8970860

**Published:** 2022-06-10

**Authors:** Wenjun Liu, Yuqiang Ji, Weiwei Zhang, Fei Fang, Qin Cai, Ying Li

**Affiliations:** ^1^Department of Cardiology, Xi'an First Hospital, Xi'an 710002, China; ^2^Central Laboratory, Xi'an First Hospital, Xi'an 710002, China; ^3^Xi'an First Hospital, Xi'an 710002, China

## Abstract

**Objective:**

To investigate the correlation between CML, sRAGE, and esRAGE and the measure of atherosclerosis of coronary heart disease.

**Methods:**

From June 2019 to December 2021, there were 100 patients in all suffering from coronary heart disease (CHD) selected as the observation group. On the basis of Gensini score, they were divided into mild group (Gensini score < 12 points), moderate group (12 points ≤ Gensini score ≤60 points), and severe group (Gensini score > 60). Apart from that, 50 normal people staying in our hospital for physical examination were chosen as the control group in the meantime. N in each group was detected and compared *ε*-Carboxymethyl lysine (CML), soluble advanced glycation end product receptor (sRAGE), and endogenous secretory advanced glycation end product receptor (esRAGE). *Pearson* correlation coefficient was adapted to assay the relevance between CML, sRAGE, and esRAGE, as well as the degree of atherosclerosis in CHD. Receiver operator characteristic (ROC) curve was applied to during the evaluation of the diagnosis of CML, sRAGE, and esRAGE, as well as their combined detection of severe atherosclerosis in CHD.

**Results:**

In contrast with the control group, the level of serum CML together with sRAGE in the observation group was considerably elevated, while the level of esRAGE appeared in a downward trend (*P* < 0.05). The level of serum CML and sRAGE was directly proportional to the measure of atherosclerosis in CHD, while the level of esRAGE was inversely proportional to the measure of atherosclerosis in CHD (*P* < 0.05). That is to say that serum CML and sRAGE were positive in matter of the measure of atherosclerosis in CHD, while esRAGE negatively appertains to the measure of atherosclerosis in CHD (*P* < 0.05). Serum CML, sRAGE, and esRAGE could effectively diagnose severe atherosclerosis in CHD, and the combined detection sensitivity (89.79%), specificity (77.16%), accuracy (86.12%), positive predictive value (86.63%), negative predictive value (88.59%), and area under ROC curve (AUC) (0.924) were higher (*P* < 0.05).

**Conclusion:**

CML and sRAGE, as well as esRAGE, are bound up with the degree of atherosclerosis in CHD, which is conducive to clinical diagnosis and treatment.

## 1. Introduction

Coronary heart disease (CHD) is widely reputed as a common or frequently occurring disease in clinical practice, which refers to the coronary artery occlusion or stenosis due to atherosclerosis, giving rise to myocardial hypoxia, ischemia, or even necrosis. The majority of clinical manifestations are chest tightness, chest pain, and aggravation after activities, which seriously threaten human health and life safety [1, 2]. There are many influencing factors of CHD, such as imbalance of lipid metabolism, diabetes, and hypertension. Currently, studies have confirmed that atherosclerosis is the basis of CHD and is a chronic pathological change caused by inflammatory response, stress response, and other reasons [3, 4]. As a consequence, it is of grand significance to investigate the pathogenesis mechanism of atherosclerosis and to assess its severity of clinical diagnosis and the effectiveness of the treatment of CHD.

At present, serological examination has become a common method of clinical examination, which is simple to operate. In addition, as a noninvasive operation, *Nε*-carboxymethyl lysine [*Nε*-(carboxymethyl) Lysine, CML], as the end product of glycation, is able to give promotion to the delivery of inflammatory factors by binding to its receptors, aggravating oxidative stress response, and ultimately aggravating atherosclerosis [5]. Studies have proven that the emergence and evolution of atherosclerosis are strongly linked with the chronic accumulation of glycosylated end products [6]. Advanced glycation end-products' (AGEs) specific receptor is a receptor for advanced glycation end products (RAGE). The soluble receptor for advanced glycation end products is soluble for RAGE, endogenous secretory receptor for advanced glycation end product (esRAGE), and endogenous secretory receptor for advanced glycation end product (sRAGE). Therefore, it is speculated that sRAGE, esRAGE, and atherosclerosis may also be related [7, 8]. However, there are few studies on the correlation between CML, sRAGE, esRAGE, and CHD atherosclerosis, which deserve further study in the future. As a consequence, the major content of the study is the exploration of the correlation between CML, sRAGE, and esRAGE and the degree of atherosclerosis in CHD, aiming to offering much more reference value to the realm of clinical diagnosis and means of treating of atherosclerosis in CHD.

## 2. Data and Methods

### 2.1. General Information

From June 2019 to December 2021, there were 100 patients in all who suffered from coronary heart disease (CHD) and were selected as the observation group to undergo coronary angiography (CAG), and the degree of coronary atherosclerosis was evaluated by Gensini score [9]. The observation group was further divided into mild group (29 cases) (Gensini score < 12 points), moderate group (39 cases) (12 points ≤ Gensini score ≤60 points), and severe group (32 cases). In addition, 50 normal people staying in our hospital for physical examination were chosen as the control group in the meantime. This study has acquired permission from the hospital ethics committee. There were no statistically significant differences in gender, age, body mass index (BMI), or family history in the matter of CHD among all participants (*P* > 0.05), and comparability has been represented in Table 1.

### 2.2. Criteria for Inclusion and Exclusion

Inclusion criteria: ① after the completion of the CAG examination, the observation group was diagnosed with CHD with no exception; ② participants with complete clinical data; ③ participants whose liver and kidney function are normal; ④ age >18; ⑤ informed consent was passed to and authorized by patients or their families.

Exclusion criteria: ① subjects with immunity, acute and chronic infections, blood diseases, etc.; ② patients who are sick for refractory hypertension, arrhythmia, valvular heart disease, congenital heart disease, myocardial disease, etc.; ③ subjects with malignant tumor; ④ subjects with severe aortic stenosis, coronary arteritis, and other diseases that can cause nonatherosclerotic coronary artery illness; ⑤ females who are pregnant or in the lactation period.

### 2.3. Detection Method

When it came to the morning after participants joining in the study, 4 mL of absolute diet venous blood was drawn from the elbow and put in an EP tube. Stewing one hour at indoor temperature, the blood samples were centrifuged for 10 min at 3000 rmp using a vm-1400-2 kb centrifuge; then, the serum was separated and stored at −80°C for the further testing. The level of CML was detected by enzyme-linked immunosorbent assay (ELISA), sRAGE, and esRAGE in serum. The kit was supplied by Shanghai Haling Biotechnology Co., LTD.

### 2.4. Observation Indicators

① Different levels of serum CML and sRAGE, as well as esRAGE, were put into comparison between two groups. ② The levels of serum CML and sRAGE, as well as esRAGE, in different atherosclerosis invalids of the observation group were put into comparison. ③ The interdependency between serum CML, sRAGE, and esRAGE levels and the measure in atherosclerosis in CHD was analyzed. ④ The merit of diagnosis of serum CML and sRAGE, as well as esRAGE levels, and their combined detection for severe atherosclerosis in CHD was analyzed.

### 2.5. Statistical Methods

SPSS 18.0 was adapted for the statistical analysis. The measurement data were in the expression as mean ± standard deviation (±*S*) and tested by *T*. Enumeration data were in the expression by example (*n*) or percentage (%) and tested by *χ*^2^. Comparison between multiple groups was performed using the *F* value. Pearson correlation coefficient was taken advantage of to investigate the association between CML, sRAGE, and esRAGE, as well as atherosclerosis degree, in CHD. Receiver operator characteristic (ROC) curve was applied to evaluate the merit of diagnosis of CML, sRAGE, and esRAGE, as well as their combined detection for severe atherosclerosis in CHD. *P* < 0.05 indicated that the differences were statistically significant.

## 3. Results

### 3.1. Contrast among Serum CML and sRAGE as wll as esRAGE Levels between Two Setting Groups

The levels of serum CML and sRAGE of the observation group were considerably in a more heightened state than those in the other one; however, the levels of serum esRAGE were considerably lower than those in the other group, with statistical significance (*P* < 0.05), which was emerged in Table 2.

### 3.2. Comparison of Serum CML and sRAGE as well as esRAGE Degrees among Different Atherosclerosis Patients of the Observation Group

The level of serum CML and sRAGE in the moderates as well as those in severe situation was considerably higher than that in mild group, and the level of serum esRAGE was considerably lower than that in mild one, while the level of serum CML and sRAGE in the severe group was considerably higher than that in moderate one, and the level of serum esRAGE was considerably lower than the control group. *P* < 0.05 indicated that the distinctions were statistically significant as emerged in Table 3.

### 3.3. Analysis to the Correlation among Serum CML, sRAGE, and esRAGE Levels as well as CHD Atherosclerosis Degree

According to Pearson correlation investigation results, serum CML as well as sRAGE were significantly bounded to the measure of atherosclerosis in CHD, while esRAGE was negatively linked to the measure of atherosclerosis in CHD. *P* < 0.05 indicated that the distinctions were statistically significant as emerged in Table 4.

### 3.4. Analysis of the Value in Diagnosis of Serum CML and sRAGE as well as esRAGE Levels and Their Combined Detection for Severe Atherosclerosis in CHD

According to ROC curve analysis results, serum CML, sRAGE, and esRAGE can effectively diagnose severe atherosclerosis in CHD. The value of sensitivity, specificity, accuracy, positive predictive, negative predictive, and area under ROC curve (AUC) were considerably higher than those of single index. *P* < 0.05 indicated that the distinctions were statistically significant as emerged in Table 5.

## 4. Discussion

CHD is recognized as a common clinical heart disease in middle-aged and elderly people. It is caused by occlusion or stenosis of coronary artery lumen, which can lead to angina pectoris, heart failure, arrhythmia, and other serious complications and even threaten patients' life safety. And its mortality is increasing year by year, which is one of the important reasons for the high clinical mortality [10]. The degree of atherosclerosis is the reflection of the evolution of CHD to a certain degree [11], so it is undoubtedly essential to evaluate the measure in atherosclerosis. For the moment, CAG is widely used in clinical diagnosis of coronary atherosclerosis, but its invasive operation has limited its clinical practice. Hence, it is indispensable to seek a convenient and noninvasive detection method [12]. Relevant studies have shown that CML, sRAGE, and esRAGE participate in the development of atherosclerosis [13, 14], but few scholars shared the experience of evaluating the correlation among CML, sRAGE, and esRAGE and the measure of atherosclerosis in CHD. The outcome of this research found out that CML, sRAGE, and esRAGE were closely associated by the extent of atherosclerosis in CHD, and the reasons are analyzed as follows.

Larsen et al. [15] concluded by Cox proportional risk analysis that sRAGE was positively correlated with major cardiovascular adverse events. It was stated by Wang et al. [16] that sRAGE was in positive proportion with cardiovascular events, while esRAGE was negatively correlated with atherosclerosis. In this study, CML and sRAGE existing in the group for observation were considerably in a more heightened state than those in the control one, yet esRAGE was considerably lower than that in the group for control. CML and sRAGE were positively correlated with atherosclerosis, while esRAGE was negatively correlated with atherosclerosis, which was basically consistent with the conclusion of Larsen and Wang. Through the research, it can be indicated that the levels of CML and sRAGE were upregulated and esRAGE was downregulated in CHD atherosclerosis patients, which were closely correlated with the degree of atherosclerosis. To analyze its possible reasons, high blood sugar can increase the viscosity of blood and cause blood flow to slow down the speed, thus cause the deposition of complex carbohydrates. And it also can increase the oxidative stress reaction, cause of fibrous tissue hyperplasia and the activity of fibrinolysis system exception occurs, eventually lead to vascular smooth muscle stiffness, especially the high level of blood glucose for a long time, which can promote the arterial wall. AGEs are likely to participate in the emergence and evolution of CHD and atherosclerosis through nonreceptor-dependent pathways such as oxidative modification of LDL, glycation, promotion of extracellular matrix synthesis, and induction of matrix protein cross-linking, or by inducing inflammatory factor release and oxidative stress associated with RAGE [17]. CML, as the main structural component and antigen epitope of AGEs, is mainly accumulated in the cytoplasm of foam cells and macrophages. Therefore, with the accumulation of AGEs, the CML level is also abnormally upregulated and participates in the development of CHD coronary atherosclerosis [18, 19]. SRAGE is derived from RAGE proteolytic cleavage and selective gene splicing on the cell surface. SRAGE can competitively bind AGEs between RAGE and RAGE, block the activation of AGEs/RAGE, and then play an inhibitory effect on vascular sclerosis [20]. However, the specific mechanism is not completely clear, and relevant studies have shown that with the increase of AGEs. The manifestation of RAGE increased continuously, and the measure of sRAGE was also upregulated, so it was suggested that the upregulation of sRAGE might be a compensatory effect physically [21]. The standard of sRAGE is the reflection of the intensity of RAGE gene expression to some extent, and the increase of sRAGE compensatory activity can antagonize tissue damage and promote inflammatory response due to high mobility group protein B-1 or advanced glycation end products (AGE) [22]. EsRAGE can avoid cell damage by competitively binding glycosylated end products and is a protective factor for vascular structure and function [23]. Currently, it has been confirmed that AGEs are strongly correlated with the emergence and evolution of CHD [24]. RAGE is a transduction receptor of AGEs' transmembrane signal and an important member of immunoglobulin superfamily receptor, which can be expressed in endothelial cells and produce various pathological effects by binding various ligands. SRAGE and esRAGE are both RAGE incomplete structures, which can competitively bind AGE with RAGE to inhibit cell signal transduction induced by RAGE, thus inhibiting vascular injury in the AGD-RAGE system [25]. Therefore, it is suggested that the degree of atherosclerosis in CHD can be judged by detecting the standard of CML and sRAGE, as well as esRAGE, and the progression of atherosclerosis in CHD can be delayed by downregulating the levels of CML and sRAGE and upregulating the levels of esRAGE.

In addition, this study found that CML, sRAGE, and esRAGE can diagnose severe atherosclerosis in CHD to a certain extent, but the detection of a single indicator has certain boundedness, as a result of which the assemble of multiple indexes was put into consideration. The results demonstrated that the accuracy, sensitivity, and specificity of the combined diagnosis of CML, sRAGE, and esRAGE were considerably higher than that in the single index. It indicated CML, sRAGE, and esRAGE could be used to diagnose severe atherosclerosis in CHD, and the mixed diagnosis of CML, sRAGE, and esRAGE was of higher value. It is suggested that multiple indexes should be combined to provide more scientific and accurate reference for clinical diagnosis and treatment.

The limitation occurred is that the impact of smoking, alcohol expenditure, diabetes, and hypertension on serum CML, sRAGE, and esRAGE indexes are not taken into account. Therefore, more comprehensive consideration is needed to obtain more scientific and accurate research results in the later stage.

In conclusion, CML, sRAGE, and esRAGE are strongly relevant to the extent of atherosclerosis in CHD. At the same time, it can also diagnose severe atherosclerosis in CHD, which is of high clinical reference value.

## Figures and Tables

**Table 1:** Comparison of general data of each group.

General information		Control group (*n* = 50)	Mild group (*n* = 29)	Moderate group (*n* = 39)	Severe group (*n* = 32)	*F*	*P*
Gender (*n* (%))	Male	27 (54.00)	16 (55.17)	21 (53.85)	17 (53.13)	0.023	0.887
	Female	23 (46.00)	13 (44.83)	18 (46.15)	15 (56.87)		
Average age (years)		59.96 ± 9.84	60.33 ± 9.80	60.04 ± 9.20	59.90 ± 9.37	0.372	0.708
Average BMI (kg/m^2^)		23.32 ± 2.90	23.04 ± 3.06	23.24 ± 3.10	23.07 ± 3.04	0.459	0.639
CHD family history (*N* (%))	Yes	4 (8.00)	2 (6.90)	3 (7.69)	2 (6.25)	0.473	0.492
	No	46 (92.00)	27 (93.10)	36 (92.31)	30 (93.75)		

**Table 2:** Contrast among serum levels of CML, sRAGE, and esRAGE between the control group and the observation group (±*s*).

Indicators	Control group (*n* = 50)	Observation group (*n* = 100)	*t*	*P*
CML (ng/mL)	389.42 ± 58.27	475.33 ± 69.45	18.195	0.000
sRAGE (pg/mL)	473.69 ± 114.36	759.68 ± 145.59	18.474	0.000
esRAGE (ng/mL)	0.45 ± 0.08	0.29 ± 0.11	9.434	0.000

**Table 3:** Comparison of serum levels in CML and sRAGE, as well as esRAGE, among invalids with different atherosclerosis in the observation group (±*s*).

Indicators	Mild group (*n* = 29)	Moderate group (*n* = 39)	Severe group (*n* = 32)
CML (ng/mL)	403.81 ± 53.16	457.16 ± 65.04^*∗*^	564.70 ± 78.35^*∗*#^
sRAGE (pg/mL)	526.08 ± 135.63	710.59 ± 152.06^*∗*^	862.49 ± 174.25^*∗*#^
esRAGE (ng/mL)	0.37 ± 0.07	0.26 ± 0.09^*∗*^	0.16 ± 0.06^*∗*#^

*Note.* Contrast with mild group, ^*∗*^*P* < 0.05; contrast with the moderate group, ^#^*P* < 0.05.

**Table 4:** Correlation among serum levels of CML and sRAGE as well as esRAGE and the degree of atherosclerosis in CHD.

Indicators	Mild group (*n* = 29)		Moderate group (*n* = 39)		Severe group (*n* = 32)	
	*r*	*P*	*r*	*P*	*r*	*P*
CML	0.393	0.001	0.327	0.018	0.430	0.000
sRAGE	0.366	0.004	0.244	0.026	0.291	0.021
esRAGE	−0.347	0.007	−0.433	0.000	−0.324	0.009

**Table 5:** Analysis to serum levels of CML, sRAGE, and esRAGE and their combined detection in the diagnosis of severe atherosclerosis in CHD.

Indicators	Optimum limit value	Sensitivity (%)	Specificity (%)	Accuracy (%)	Positive predictive value (%)	Negative predictive value (%)	AUC	95% CI
CML	538.07 (ng/mL)	59.02	72.34	63.19	62.36	73.44	0.706	0.599∼0.803
sRAGE	785.83 (pg/mL)	56.46	74.75	61.68	65.36	61.30	0.670	0.557∼0.774
esRAGE	0.18 (ng/mL)	82.10	77.16	71.68	70.94	77.33	0.827	0.818∼0.943
Joint detection	—	89.79	77.16	86.12	86.63	88.59	0.924	0.869∼0.968

*Note.* Compared with CML, sRAGE, and esRAGE, ^*∗*^*P* < 0.05.

## Data Availability

The data used to support the findings of this study are available from the corresponding author upon request.
